# Block of Proliferation 1 Promotes Proliferation, Invasion and Epithelial Mesenchymal Transformation in Gastric Cancer

**DOI:** 10.1155/2022/2946989

**Published:** 2022-02-16

**Authors:** Jing He, Ziwei Chen, Qingfeng Xue, Wenyu Shi

**Affiliations:** ^1^Department of Chemotherapy, Affiliated Hospital of Nantong University, Nantong, China; ^2^Research Center of Clinical Medicine, Affiliated Hospital of Nantong University, Nantong, China; ^3^Department of Cardiology, Affiliated Hospital of Nantong University, Nantong, China; ^4^Department of Oncology, Affiliated Hospital of Nantong University, 20 Xisi Road, Nantong, China

## Abstract

**Background:**

Gastric cancer (GC) is one of the leading causes of cancer-related death worldwide nowadays. Block of proliferation 1 (BOP1), a nucleolar protein involved in rRNA processing and ribosome assembly, is associated with tumor development in certain cancers of digestive system. Therefore, we hypothesized that BOP1 might play an important role in gastric cancer development.

**Methods:**

Gene Expression Omnibus (GEO) database and The Cancer Genome Atlas (TCGA) were used to identify the differentially expressed genes and their clinical relevance. qPCR and western blot were performed further to examine the levels of BOP1 mRNA and protein, respectively. Cell viability, apoptosis, migration and invasion were investigated in gastric cancer cell lines with BOP1 silencing or overexpression. The epithelial mesenchymal transition (EMT) associated proteins, including E-cadherin and N-cadherin, were measured using immunoblotting. Finally, the downstream pathway of BOP1 were explored using bioinformatic analysis and qPCR.

**Results:**

BOP1 was found up-regulated in gastric tumor tissues compared with paired normal tissues (P < 0.0001). Its expression was associated with more advanced pathological grades (P = 0.0006) and tumor location (P = 0.002), as well as a poor survival (HR 1.27, P = 0.015). BOP1 expression was increased in 4 kind of tumor cell lines compared with the normal group. The overexpression of BOP1 promoted cell proliferation and inhibit cell apoptosis, while silencing BOP1 showed a reversed trend. Immunoblotting results suggested that BOP enhanced N-cadherin, a mesenchymal marker, while reduced E-cadherin, an epithelial marker. Finally, bioinformatic prediction showed that the cell cycle could be a downstream pathway of BOP1.

**Conclusions:**

The present study demonstrated that BOP1 contributed to the development of gastric cancer by promoting proliferation, invasion and epithelial mesenchymal transformation, which could be a biomarker or therapeutic target in GC.

## 1. Introduction

Gastric cancer (GC) is the leading cause of morbidity among digestive system malignancy. It is the second cause of cancer-related death worldwide, claiming 723000 lives every year [1, 2]. The contributing factors include helicobacter pylori, nitrite intake and chronic gastric diseases. However, due to lack of typical symptoms and signs during the early phase, the majority of patients were diagnosed at advanced stage, accompanied by metastasis to lymph node and distant organs [3]. Meanwhile, current therapies such as chemotherapy, immunotherapy, and molecular target therapy are not effectively. Considering the poor prognosis gastric cancer, it is necessary to further explore the molecular mechanism of GC.

The protein Block of proliferation 1 (BOP1), a member of PES1-BOP1-WDR12 complex, regulates the maturation of 5.8S/28S rRNA and biogenesis of 60S ribosomal subunits [4, 5]. Mechanically, BOP1 is located in the pre-60S ribosomal complexes, and responsible for rRNA maturation and biogenesis when recruiting PES1 [6]. The balance between ribosome biogenesis and cellular division is vital for cell growth, whose dysregulation can cause the cell cycle arrest [7, 8]. Besides, BOP1 was reported to influence cell cycle by modulating P53 accumulation [9, 10]. Recently, BOP1 played an oncogenic role in the hepatocellular carcinoma (HCC) and melanoma. BOP1 can promote the process of epithelial mesenchymal transformation in HCC and mediate BRAF inhibitor resistance in melanoma [11, 12]. However, the specific role of BOP1 in the gastric cancer has not been investigated.

Therefore, our study aimed to study the effect of BOP1 on proliferation and metastasis of gastric cancer cells and the possible downstream pathway, which could be a biomarker or therapeutic target in gastric cancer.

## 2. Methods and Materials

### 2.1. Cell Culture

Human gastric epithelial cell line (GSE-1) and gastric cancer cell lines (HGC27, N87, MGC803 and BCG823) were purchased from American Type Culture Collection (ATCC) and were cultured in the DMEM/F12 supplemented with 1% penicillin/streptavidin and 10% FBS (Gibco; USA). The cells were cultured in a humidified atmosphere of 37°C containing 5% CO2.

### 2.2. Bioinformatic Analysis

NCBI-Gene Expression Omnibus database (GEO) (https://www.ncbi.nlm.nih.gov/) is a public database containing microarray and high throughput sequencing. Both GSE103236 and GSE118916 are microarrays containing tumor and adjacent normal tissues based on the platforms GPL4133 (Agilent-014850 Whole Human Genome Microarray 4x44K G4112F) and GPL 15207(Affymetrix Human Gene Expression Array). 5 pairs were selected randomly for further analysis. Clinical features **of** gastric cancer were extracted from the cancer genome atlas (TCGA) database. By integrating all the expression profiles, we conducted the survival analysis, Gene Ontology (GO), Kyoto Encyclopedia of Genes and Genomes (KEGG) analysis. The differently expression genes were identified by utilizing the limma package in R programme, with the cut-off criterion of |Fold change| > 2 and P Value <0.01.

### 2.3. RNA Extraction and Quantitative Real Time PCR Assay

Total RNA was extracted from cultured cells by using the Trizol reagent (Invitrogen) according to the manufacturer's instructions. Purity of RNA was tested using the Nanodrop and RNA was cleaned up with an DNAse-digested and RNeasy Kit (Qiagen) to prevent the DNA contamination. Then, 1000 ng RNA was transcribed into cDNA by a commercial kit (TaKaRa, Japan). Quantitative real time PCR assays was conducted using a SYBR Premix Ex Taq kit (Takara, Japan) according to the manufacturer's instructions. All the experiments were performed for three times.

### 2.4. Cell Transfection

The human BOP1 overexpression vector and si-BOP1 expression vector were purchased from GenePharma (Shanghai, China). pcDNA3.1 vector containing full length BOP1 and two si-BOP1 vectors were transfected using Lipofectamine 2000 (Thermo, USA). The overexpression and knockdown efficiency were measured by quantitative real time PCR.

### 2.5. Western Blot

All the cells were collected 72 hours after transfection. Protein sample was separated by SDS-PAGE gel electrophoresis and transferred to the nitrocellulose filter membrane by semi-dry conversion, followed by blocked with a 5% fat-free milk. The primary antibodys were incubated at the dilution of 1 : 1000 overnight, followed by secondary antibody. The bands were visualized using the enhanced chemiluminescence detection kit (Thermo, USA).

### 2.6. Wound-Healing Assay

Cells were cultured in a 6-well plate and scratched for a straight wound. The process of cell migration was imaged after 24 hours. The wound healing was calculated as (0-hour width-24-hours width)/0-hour width x 100%.

### 2.7. Cell Invasion Assay

Cell invasion was evaluated using 8-*μ*m pore size transwell chambers (Corning, USA). Cells were plated in the upper chamber and completed medium was added as a chemoattractant in the lower chamber. The upper chamber was coated with 30 *μ*g of Matrigel (BD Biosciences, USA). After 24 hours of incubation, cells entering the lower chamber were fixed in the 4% paraformaldehyde and stained with crystal violet. We randomly selected five microscopic fields to count the cell number and captured the images under the microscope.

### 2.8. Cell Viability Assay

The tumor cells were cultured in 96-well flat-bottomed plates. 10 *μ*L CCK-8 solution (Beyotime, China) was added to each well at different time points post transfection (0, 12, 24, 36, 48, 60, and 72 h). After 4 hours incubation, a microplate reader was utilized to evaluate the optical value (OD) at 450 nm of absorbance. We conducted this experiment in 6 independent replicates.

### 2.9. Flow Cytometer Analysis

Tumor cells (2 × 10^5^ cell/well) were collected in 200 *μ*L Annexin V binding buffer (Beyotime, China) and 20 *μ*L Annexin V/propidium iodide (PI) reagent in the dark. The proportion of apoptosis was measured by FACSCalibur flow cytometer (BD Biosciences, USA).

### 2.10. Statistical Analysis

Statistical analyses were performed using Prism 8.0 (GraphPad, USA). All the experiments were conducted in at least three biological replicates and data were expressed as mean ± s.e.m. Student's t-test was applied to compare between two groups and one-way ANOVA was used for more than two groups. The *χ* 2 -test was conducted to analyze the impact of race, gender, HP infection, T, N, M stages on the BOP1 expression in TCGA human samples. P value <0.05 was considered statistically significant.

## 3. Results

1. BOP1 was upregulated in gastric cancer and related to the metastatic ability

We performed differentially expressed gene analysis based on two GEO profile, and identified 26 common genes with the criterion of |log2 fold change| > 2 and P < 0.01 (Figure 1(a); Table 1). Then, we constructed heat map and volcano map to visualize these genes between gastric tumor samples and paired normal tissues (Figure 1(b) and 1(c)). Among them, BOP1 is up-regulated gene and is associated with digestive cancers. In addition, BOP1 expression was upregulated in TCGA database when comparing tumors tissues to the corresponding normal tissues (Figure 1(d), P< 0.0001). We also BOP1 expression is related to more advanced pathological grades (Figure 1(e), P = 0.0096) and tumor sites (Figure 1(f), P = 0.0272). While tumor weight did not correlate with BOP1 level (Figure 1(g), P = 0.2393). We grouped patients from TCGA database as two groups according to the quartile of expression of BOP1 and analyzed the relationship between BOP1 expression and clinical parameters. As indicated in Table 2, we found that lymph node metastasis was closely associated with BOP1 expression while no significant correlations were observed between other clinical parameters and BOP1 expression. These results suggested that BOP1 might participate in the occurrence and metastasis of gastric cancer.

(2) BOP1 predicted poor prognosis in gastric cancer patients

We performed Kaplan–Meier survival analysis to assess the overall survival by pooling the data of 876 patients from Kaplan-Meier Plotter database. Higher expression of BOP1 was related to poor overall survival in patients with gastric cancer (HR, 1.27; 95% CI, 1.05-1.53; P < 0.05) (Figure 2(a)). The overall survival was not different in gastric cancer with moderate and well differentiated (Figure 2(b) and 2(d)), but in poorly differentiated grade (HR, 1.95; 95% CI, 1.31-2.92; P < 0.001) (Figure 2(c)).

(3) BOP1 promotes proliferation and inhibits apoptosis in GC cells

We have detected the expression of BOP1 mRNA and protein in a normal gastric epithelial cell line (GSE-1) and 4 tumor cell lines (HGC-27, N87, MGC-803 and BCG-823). It showed that all tumor cell lines had higher BOP1 mRNA expression than GSE-1 cells (Figure 3(a)). Immunoblotting results also showed that BOP1 protein was highly expressed in HGC-27 and MGC-803 (Figure 3(b)). Considering that HGC-27 had the highest while N87 had the lowest expression level of BOP1, we knocked down BOP1 in the HGC-27 cell line and overexpressed it in the N87 cell line (Figure 3(c) and 3(d)). Malignant tumors are characterized by excess proliferation and resistant apoptosis. Cell viability and apoptosis assay showed that BOP1 could enhance proliferation and inhibit apoptosis in GC cells (Figure 3(e) and 3(f)). Immunoblotting results also showed BOP1 increased the expression of p21 and cleaved caspase 3 (Figure 3(g)). Taken together, our findings suggested the oncogenesis role of BOP1 in the gastric cancer.

(4) BOP1 promotes epithelial mesenchymal transformation (EMT) in GC cells

EMT progression is of great significance in gastric cancer accompanied by distant metastasis [13]. As indicated in Figure 4(a) and 4(b), BOP1 overexpression enhanced the migratory and invasive capacity of N87 cells. While silencing BOP1 showed a reversed trend in HGC-27 cell line. Then, we detected the protein level of E-cadherin and N-cadherin and found BOP1 could upregulate N-cadherin while downregulate E-cadherin (Figure 4(c)). Collectively, these finding suggested BOP1 was a possible driver for the tumor metastasis.

(5) The prediction of downstream biological process affected by BOP1

To further explore the role of BOP1 in the oncogenesis and metastasis in the gastric cancer, we tried to figure out some potential biological process that might be modulated by BOP1. We selected 20 patients from the GEO database divided them into hi-BOP1 and low-BOP1 group according to the expression of BOP1 and performed differentially expression analysis with |log2 fold change| >1 and P < 0.001. Totally, 78 differently expressed genes were identified and visualized by volcano map (Figure 5(a)). Then, we performed GO analysis (Figure 5(b)) and KEGG analysis (Figure 5(c)) to explore the enriched pathways that BOP1 might participate in. The differentially expressed genes were involved in cell division and cell cycle. Besides, the expression of CKDN2B, CKDN1A and CKDN1B, as the suppressors of cell cycle, were significantly downregulated in cells with high BOP1 expression (Figure 5(d)), suggesting that cell cycle could be modulated by BOP1. However, Further experiments should be performed to explain the underlying mechanisms.

## 4. Discussion

In our study, we investigated for the first time the effect of block on proliferation 1 (BOP1) on gastric cancer. We found that BOP1 was significantly upregulated in the GC tissues and cell lines. Further, overexpression of BOP1 could promoted cell proliferation and inhibit cell apoptosis in GC cell lines. However, silencing BOP1 showed a reversed trend. Besides, BOP1 was found to promote cell invasion in GC through regulating the EMT process [13]. Finally, we preliminarily explored the potential downstream biological targets of BOP1 using genomic bioinformatics, and found that BOP1 could affect cell cycle pathway.

BOP1, located on 8q24, is a WD40 protein and was isolated from embryonic fibroblasts initially [14]. Due to the close location to MYC gene in the chromatin and its role in rRNA processing, some studies have explored the function of BOP1 in some malignancies. BOP1 was found overexpressed in the colorectal tumor tissues and its expression level was related with copy number variation of MYC [15]. BOP1 was found upregulated in the ovarian tumor and related to strong methylation [16]. Besides, BOP1 was reported to influence the epithelial mesenchymal transformation in hepatocellular carcinoma (HCC) through upregulating F-actin, c-catenin and vimentin, which was similar to our findings in the GC cell lines [12]. Taken together, previous findings in other malignancy supported our exploratory study of BOP1 function in gastric cancer.

rRNA maturation process and ribosomal biogenesis are currently considered as important process in the oncogenesis and development in tumors. In cancer therapy, chemical reagents targeting multiple steps in rRNA transcription have been proved effective in killing tumors [17, 18]. Ribosomes are indispensable to translate mRNA into functional protein. While the disturbance of ribosome may lead to the accumulation of dysfunctional proteins [19–21]. Besides, Ribosomal biogenesis is the biological process in need of large sum of energy in human cells. The impaired ribosomal biogenesis cannot meet the growth needs of cancer cells thus limit the proliferation [22]. Some studies have confirmed that hyperactive ribosome biogenesis can accelerate tumor progression and malignant transformation through stabilizing P53 [23–25]. Our study also confirmed that BOP1 could promoted gastric cell proliferation and invasion by regulating cell cycle.

However, some limitations existed in our study. For example, the specific downstream molecular targets and pathways were not identified. Besides, some in vivo experiments were not conducted. In the future, more experiments warranted further explanation of BOP1 in GC.

## 5. Conclusion

In summary, we have described the oncogenic role of block on proliferation 1 (BOP1) in gastric cancer and found that BOP1 promoted cell proliferation, invasion and EMT. Our results suggested that BOP1 could serve as a novel molecular target for GC treatment.

## Figures and Tables

**Figure 1:** BOP1 was up-regulated in gastric cancer (GC) and was associated with pathological grades based on online databases. (a) A total of 26 genes were differentially expressed (fold change>2 and P < 0.01) between tumor tissues and the adjacent normal tissues from two GEO profiles (GSE103236 and GSE118916). (b) The Heat map showed the relative expression of 26 genes in 5 paired GC tissues. (c) The Volcano map showed all differentially expressed genes. (d) BOP1 expression was compared between tumor tissues and the adjacent tissues from TCGA database(P < 0.0001). BOP1 expression was compared among (e) pathological grades (G1, G2 and G3) (P = 0.0096), (f) tumor location (antrum, fundus/body, gastroesophageal junction and cardia/proximal) (P = 0.0272). and (g) tumor weight group (P = 0.2393).

**Figure 2:** BOP1 was negatively correlated with overall survival, especially in patients with poorly differentiated tumors. (a) Kaplan–Meier survival curves were illustrated for patients with low or high level of BOP1 expression in GC (a), well differentiated GC (b), poorly differentiated GC (c), and moderately differentiated GC (d).

**Figure 3:** BOP1 promotes proliferation and inhibits apoptosis in GC cells. The expression of BOP1 mRNA (a) and protein (b) were measured in 5 different gastric cell lines including GSE-1, HGC-27, N87, MGC803 and BCG823. The expression of BOP1 mRNA (c) and protein (d) were measured in BOP1-overexpressed N87 cell and BOP1-silencing HGC-27 cell. (e) Cell viability was detected by CCK-8 in different time points (0, 24, 48, 72 and 96 hours after transfection) in HGC-27 and N87 cells. (f) The proportion of apoptotic cells were detected by flowcytometry. (g) The expression level of caspase 3 and p21 were measured. The data are expressed as the means ± s.e.m. of three experiments. (∗P < 0.05, ∗∗P < 0.01, ∗∗∗P < 0.001).

**Figure 4:** BOP1 enhanced the migration and invasion of gastric cancer cells. The N87 cell line was used to overexpress BOP1 while HGC-27 cell line was to silence BOP1. (a) The migratory capability was evaluated by wound-healing assay. (b) The invasive ability was evaluated by transwell assay. Representative images were shown and results were quantified. (c) The relative expression of N-cadherin and E-cadherin were measured in treated HGC-27 and N87 cells.

**Figure 5:** BOP1 was involved in a variety of biological processes. (a) Differentially expressed genes were shown by the volcano map in gastric tumors with high-BOP1 and low-BOP1 expression (Fold change>1, P < 0.001). (b) The differentially expressed genes were enriched by GO analysis of biological processes, and (c) KEGG pathways. (d) The genes involved in cell cycle were measured by qPCR.

**Table 1:** The differentially expressed genes in gastric cancer.

	Fold change (normal/tumor)	P.Value
Up-regulated		
VAV2	2.43E-291	0.00054296
PDCD4	1.94E-267	0.00155397
ATP11A	1.88E-256	0.00025124
DMRTA1	3.67E-252	0.00889797
KIF22	1.87E-235	0.00720126
GTPBP4	2.24E-183	0.00462927
KIT	7.51E-176	0.00123613
E2F3	4.67E-163	0.00181371
RAD51AP1	7.28E-158	0.00970767
SLC26A9	7.42E-141	0.00698115
NT5DC2	5.42E-93	0.00975628
BOP1	6.60E-90	0.00161215
ACTR5	3.13E-75	0.00636983
UBE2T	1.10E-68	0.0043718
NUP107	1.74E-41	0.00747152
Down-regulated		
ATIC	112144.551	0.00096759
PUF60	7.3161E+15	0.00801933
POLR1C	1.492E+17	0.00126633
TMEM206	1.659E+18	0.0066626
DDAH2	4.48E+29	0.00282228
NUDT5	3.07E+31	0.00634813
ERF	1.80E+41	0.00664546
TIMELESS	1.44E+65	0.00094449
HSPH1	5.23E+85	0.00773883
SPTAN1	3.11E+166	0.00187708
EZH2	5.28E+269	0.00014716

**Table 2:** The clinical characteristics according to the expression of BOP1.

Variables	BOP1 expression		
	Negative (n = 152)	Positive (n = 77)	P. Value
Age, years	64.2 ± 13.8	66.6 ± 15.9	0.1049
Sex			0.317
Male	101	46	
Female	51	31	
Race			0.060
Asian	27	27	
White	101	39	
Black	24	11	
HP infection			0.486
Yes	6	2	
No	146	75	
Vital status			0.548
Alive	110	40	
Dead	42	37	
T stage, n (%)			0.325
T1	7	6	
T2-4	145	71	
N stage, n (%)			0.002∗
N0	39	35	
N1-3	113	42	
M stage, n (%)			0.129
M0	140	66	
M1	12	11	

## Data Availability

All data could be available upon request from the corresponding author.
